# Identification of Metabolism-Related Genes Influencing Prognosis of Multiple Myeloma Patients

**DOI:** 10.1155/2021/6574491

**Published:** 2021-12-15

**Authors:** Rui Wang, Wenxuan Bu, Yang Yang

**Affiliations:** Department of Hematology, People's Hospital of Lianshui, Lianshui 223400, Huai'an, China

## Abstract

Multiple myeloma (MM) is the second most commonly diagnosed hematological malignancy. Understanding the basic mechanisms of the metabolism in MM may lead to new therapies that benefit patients. We collected the gene expression profile data of GSE39754 and performed differential analysis. Furthermore, identify the candidate genes that affect the prognosis of the differentially expressed genes (DEGs) related to the metabolism. Enrichment analysis is used to identify the biological effects of candidate genes. Perform coexpression analysis on the verified DEGs. In addition, the candidate genes are used to cluster MM into different subtypes through consistent clustering. Use LASSO regression analysis to identify key genes, and use Cox regression analysis to evaluate the prognostic effects of key genes. Evaluation of immune cell infiltration in MM is by CIBERSORT. We identified 2821 DEGs, of which 348 genes were metabolic-related prognostic genes and were considered candidate genes. Enrichment analysis revealed that the candidate genes are mainly related to the proteasome, purine metabolism, and cysteine and methionine metabolism signaling pathways. According to the consensus clustering method, we identified the two subtypes of group 1 and group 2 that affect the prognosis of MM patients. Using the LASSO model, we have identified 10 key genes. The prognosis of the high-risk group identified by Cox regression analysis is worse than that of the low-risk group. Among them, PKLR has a greater impact on the prognosis of MM, and the prognosis of MM patients is poor when the expression is high. In addition, the level of immune cell infiltration in the high-risk group is higher than that in the low-risk group. In the summary, metabolism-related genes significantly affect the prognosis of MM patients through the metabolic process of MM patients. PKLR may be a prognostic risk factor for MM patients.

## 1. Introduction

Multiple myeloma (MM) is a hematological malignant tumor derived from abnormal monoclonal plasma cells. The main clinical symptoms include anemia, infection, bone destruction, and renal insufficiency [1]. Due to the lack of specificity of these clinical symptoms for the diagnosis of MM, this has also led to the current lack of time-sensitive methods for the diagnosis of MM [2]. In recent years, with the rapid increase in the morbidity and mortality of MM, its occurrence and development factors and prognosis have gradually been paid attention to [3]. It is currently known that MM is prone to occur in middle-aged and elderly men, and the median survival time is about six years [4]. Meanwhile, the World Health Organization classification system specifically distinguishes MM from other plasma cell diseases [5]. Moreover, MM has also become the second most common hematological malignancy after non-Hodgkin's lymphoma [6]. In general, MM can be alleviated by many clinical drugs and treatment techniques, for example, high-dose chemotherapy, hematopoietic stem cell inhibition, and proteasome inhibitors (bortezomib and immunomodulator lenalidomide) [7]. However, these treatments cannot make MM patients escape the fate of disease recurrence and aggravation [8]. Therefore, exploring new therapeutic targets and disease prognostic indicators for MM is of great significance for the treatment of MM patients.

The tumor is known for its special function of promoting the unlimited proliferation of tumor cells [9]. Its particularity is partly due to the generation or inhibition of metabolites in tumor cells and the changes of metabolic pathways, which include the changes of glycolipid and protein metabolic pathways [10], which provide sufficient energy and nutrition supply for the unlimited and rapid proliferation of tumor cells [11]. In addition, changes in metabolic pathways also affect the expression of transcription factors involved in regulating tumor cell proliferation and apoptosis [12]. Therefore, understanding the metabolic changes and the upstream and downstream regulatory genes of metabolic changes in tumor cells can not only provide early warning for tumor occurrence but also provide a reference and qualitative gold standard for tumor treatment and improving the prognosis of tumor patients.

Metabolic changes are a common feature of most tumorigenesis. As a nonsolid tumor in the bone marrow, the metabolic process of MM has gradually been clarified with the deepening of research and the development of research methods. Moreover, changes in metabolic pathways also affect the efficacy of different treatment methods in MM. In this process, different targeted treatment methods are also being developed and applied. However, the diagnosis, treatment, and prognosis of MM are still trouble people. Therefore, this study intends to evaluate the impact of metabolism-related genes on the prognosis of MM patients by transcriptome sequencing and predict the risk factors of MM prognosis, in order to provide a theoretical basis for the treatment of MM patients and improve their prognosis and survival rate.

## 2. Materials and Methods

### 2.1. Data Procession

The gene expression profiles of GSE39754 were downloaded from the Gene Expression Omnibus (GEO) database. The GSE39754 included gene expression profiles of CD138 purified myeloma plasma cells from 170 newly diagnosed MM patients and 6 CD138 purified plasma cells from healthy donors. The data were analyzed with the Affymetrix package. The differentially expressed genes (DEGs) were calculated by limma package [13]. Set the filtering threshold |log2 fold change (FC)*|* > 1 and *P* < 0.05. Genes associated with the metabolism were accessed in the MSigDB database.

### 2.2. Cox Regression Analysis

The “survival” package of R was used to do the Cox single factor analysis, and then, metabolic-related genes affecting MM patient survival were then screened. Candidate genes were used to build a binomial least absolute shrinkage and selection operator regression (LASSO) model using the glmnet R package [14]. MM samples were divided into high and low-risk groups based on the median level of score in Cox multivariate regression analysis. Kaplan–Meier (KM) curves were generated to assess the prognostic value of high and low-risk groups using the survival R package.

### 2.3. Identification of MM Subtypes

The ConsensusClusterPlus package was used to cluster the expression of candidate genes in MM samples. 170 samples of GSE39754 MM were divided into two subtypes (group 1 and group 2).

### 2.4. Enrichment Analysis

Gene Ontology (GO) and KEGG pathway analysis of candidate genes were carried out by enrichGO and enrichKEGG functions of clusterProfiler package. Terms in enriched GO and KEGG pathways were identified according to the cutoff criterion of *P* < 0.05.

### 2.5. Immune Score

The CIBERSORT was used to quantify the immune infiltration level of MM through the 22 immune cells. The limma package was used to calculate the difference between high and low-risk groups.

## 3. Results

### 3.1. Differentially Expressed Genes in Multiple Myeloma

To identify gene expression abnormalities of multiple myeloma, we identified differentially expressed genes between MM and controls in GSE39754. A total of 2821 differentially expressed genes (DEGs) were identified, including 1317 upregulated and 1504 downregulated expressions (Figure 1(a)). Subsequently, we identified 576 DEGs related to the metabolism (DEMRGs) using the MSigDB database. In a Cox regression analysis of metabolism-related genes in the MSigDB database, we identified 2151 genes significantly associated with overall survival (OS) in MM. Thus, we obtained 348 DEMRGs significantly affecting OS of MM, which was identified as candidate genes (Figure 1(b)). These genes were significantly differentially expressed in MM and controls (Figure 1(c)).

### 3.2. Biological Roles Related to Candidate Genes

To identify the mechanism of action of candidate genes in MM, we performed an enrichment analysis. Results of GO showed that (Figure 2(a)) candidate genes significantly enriched in regulation of the cellular amine metabolic process, regulation of the cellular amino acid metabolic process, and regulation of mRNA stability of the biological process (BP). The ficolin-1-rich granule lumen, ficolin-1-rich granule, and cytoplasmic vesicle lumen in cellular composition (CC) were significantly enriched by candidate genes. Peptidase activity, acting on L-amino acid peptides, RNA binding, and oxidoreductase activity, acting on the CH-OH group of donors, NAD or NADP as an acceptor of molecular functions (MF) were significantly involved by candidate genes. In addition, KEGG signaling pathways enriched by candidate genes mainly included proteasome, purine metabolism, and cysteine and methionine metabolism (Figure 2(b)).

### 3.3. Identified Key Genes for Multiple Myeloma

MM samples were divided into group 1 and group 2 by candidate genes using consensus clustering (Figure 3(a)). Survival analysis results showed that patients in group 2 had better prognosis compared to group 1 (Figure 3(b)). In addition, there were differences in the expression of candidate genes in group 1 and group 2 (Figure 3(c)). It is suggested that candidate genes may differentiate MM patients by prognostic status.

To identify specific prognostic genes among the candidate genes, we performed LASSO regulation analysis. When log(*λ*) = 78 was selected, a model was developed based on a 78-gene signature in candidate genes (Figures 4(a) and 4(b)). The top 10 genes with the largest absolute values of the lasso regression coefficients were further screened as key genes. Moreover, to further evaluate the prognostic role of the key genes, we constructed nomograms using Cox regression analysis. Among the key genes, we found that downregulated PKLR contributed the most to the good prognosis of MM patients (Figure 4(c)).

### 3.4. Risk Score of Key Genes

To evaluate candidate genes, we utilized Cox regression analysis to divide the MM sample into high and low-risk groups by the median of the risk scores (Figure 5(a)). There were fewer patients with MM who ultimately survived in the high-risk group compared with the low-risk group. The expression of candidate genes differed in the high-risk and low-risk groups. Among them, the higher the expression of PKLR, the worse the prognosis of MM patients. In addition, the risk score had a good predictive ability for the prognosis of patients with MM (AUC > 0.6) (Figure 5(b)). The overall survival probability was significantly lower in the high-risk group than in the low-risk group (Figure 5(c)).

### 3.5. Immune Infiltration in Multiple Myeloma

The method of CIBERSORT was applied to detect 22 immune cell infiltration levels in high-risk and low-risk groups of MM (Figure 6(a)). Differential analysis revealed that CD4+ T cell memory resting, NK cell resting, monocyte, macrophage M0, eosinophil, and neutrophil had higher infiltration levels in the high-risk group, while B cell plasma had lower infiltration levels in the high-risk group, compared with the low-risk group (Figure 6(b)).

## 4. Discussion

In this study, 348 metabolism-related prognostic genes were identified. Further studies showed that the candidate genes were mainly related to the proteasome, purine metabolism, and cysteine and methionine metabolism. In addition, the expression of PKLR was significantly different between the high-risk group and the low-risk group, suggesting that the expression of PKLR plays a regulatory role in the prognosis of MM.

In the process of tumor, many kinds of cell processes changed in tumor cells of MM. MM tumor cells multiply rapidly and accelerate the tumor process, which will inevitably lead to changes in some traits in tumor cells. Genes are the individual units that regulate characteristics, and their expression levels also determine the differences in tumor cell characteristics. In addition, in order to meet the needs of cell proliferation in tumor cells, the changes in their metabolic levels must also be regulated by metabolism-related genes. The study of metabolism-related genes can enable us to better understand the occurrence of tumor cells and promote the treatment of tumors, which is of great significance. In this study, 2821 DEGs were identified, of which 576 DEGs are related to the metabolism. Research on these DEGs may have a certain effect on the treatment of MM.

Further analysis of 576 DEGs in MM. We found that these DEGs are mainly enriched in the process of regulating the amino acid metabolism. Amino acid metabolism disorder is an important indicator of tumorigenesis [15]. The uptake of amino acids by tumor cells through the tumor microenvironment can not only provide raw materials for nitrogen and carbon sources of protein and nucleotide for proliferation but also help to maintain the carbon metabolism and redox reaction in tumor cells [16, 17]. In the current research on the amino acid metabolism of MM, glutamine is known to play an important role in the process of MM. Glutamine that enters the cell can be broken down into glutamate and amines. This has also become a marker of the process of MM. Marina et al.' study showed that the feasibility of this method was confirmed by drawing bone marrow and detecting the expression of glutamate and amine [18]. Meanwhile, inhibiting the intake of glutamine may provide a new strategy for the treatment of MM [18]. In addition, changes in the methionine metabolism also play an important role in tumor progression. Gao et al. [19] found that restricting methionine intake in cancer patients can improve the occurrence and development of tumors. However, research on the effect of changes in the methionine metabolism on MM is relatively rare. In this study, DEGs are enriched in the methionine metabolic pathway, which indicates that the methionine metabolic pathway plays an important role in the occurrence and development of MM. Meanwhile, the study showed that cysteine is a key amino acid for the survival of tumor cells. Depletion of cysteine in mice using cysteinase can promote iron death of tumor cells [20]. Meanwhile, Nunes et al. [21] have also proved that the level of cysteine in blood can be used as a detection indicator for cancer. In the study, DEGs are also enriched in the molecular functions of peptidase active and acting on L-amino acid peptides. Moreover, KEGG analysis also showed that these differential genes are enriched in the cysteine and methionine metabolism, which further suggests that the occurrence of MM is related to the amino acid metabolism.

Due to the abnormal chromosomes of tumor cells, the large and rapid proliferation will also lead to excessive protein synthesis [22]. The selective degradation of excess protein plays an important role in the development of cancer. The abundant proteasomes play a major role in the protein degradation process of cancer [23]. The high expression of the proteasome in MM has been reported [24]. Meanwhile, the proteasome also has the role of cancer antigen production and presentation, which is also an indispensable condition for immune surveillance and tumor treatment [22, 25]. Therefore, artificial intervention in the expression of proteases in MM cells is of great significance for the treatment of tumors. In this study, metabolism-related DEG is enriched in the proteasome metabolic pathway, which indicates that the proteasome plays an important role in the occurrence of MM. This also further confirmed the role of the aforementioned proteasome in MM.

## 5. Conclusion

Glycolysis is a reaction system for tissue cells in the body to maintain normal physiological functions and provide energy [26]. In the cancer process, a variety of important functional enzymes in the glycolysis process are strengthened to produce more energy, and its glycolysis metabolite lactic acid can also provide energy for tumor cells in a series of fermentation processes [27]. This feature of glycolysis is also valued in prognostic testing of cancer patients [28]. Then, there are a wide variety of genes and enzymes involved in glycolysis [29]. Researchers have also screened different genes and key enzymes in the glycolysis process through different research methods to predict prognostic conditions [30]. Regrettably, there is still no gold standard for a good prognosis in the process of glycolysis. In this study, we screened the metabolic-related DEGs and found that the higher the expression of PKLR, the worse the prognosis of MM, which indicated that PKLR had a better diagnostic value in the prognosis diagnosis.

In summary, MM differentially expressed genes are mainly enriched in metabolic signaling pathways. Further research shows that PKLR can be used as a key marker for the prognosis of MM.

## Figures and Tables

**Figure 1:** Identification of metabolism-related differentially expressed genes in multiple myeloma. (a) Volcano plot of differentially expressed genes between MM and controls. Red is upregulation and green is downregulation. (b) Intersection of genes affecting MM survival and metabolism-related differentially expressed genes. (c) Expression heatmap of candidate genes in MM and control samples. MM, multiple myeloma.

**Figure 2:** Enrichment analysis of candidate genes. (a) The main GO results of candidate genes enriched. (b) The main KEGG pathways of candidate genes enriched.

**Figure 3:** Identification of new subtypes of multiple myeloma. (a) Consistency clustering analysis conducted according to DEMRGs. (b) Differences in overall survival between MM patients of group 1 and group 2. (c) Clustered heatmap of genes in group 1 and group 2.

**Figure 4:** Identification of key diagnostic genes for multiple myeloma. (a) Selection of optimal parameter (*λ*) in the LASSO model. (b) LASSO coefficient profiles of 78-gene signature. (c) Nomogram to predict the prognosis of MM.

**Figure 5:** Risk score analysis of key genes in multiple myeloma. (a) Risk score and survival status distribution according to the median of the risk score for each key gene. (b) ROC curves of risk scores to predict patients' 1 and 3-year survival. (c) Kaplan–Meier survival curves of MM patients for high and low-risk groups.

**Figure 6:** Immune cell infiltration in high and low-risk groups. (a) Heatmap of immune cell infiltration in high and low-risk groups of multiple myeloma. (b) Differences in infiltration of immune cells between high and low-risk groups.

## Data Availability

The datasets used and/or analyzed during the current study are available from the corresponding author upon request.
